# A Social-aware and Mobile Computing-based E-Commerce Product Recommendation System

This article has been retracted.

**DOI:** 10.1155/2022/9501246

**Published:** 2022-03-19

**Authors:** Qin Xu, Jun Wang

**Affiliations:** ^1^Department of Economics and Management, Wuhu Institute of Technology, Wuhu 241003, China; ^2^Department of Information Construction and Management, Wuhu Institute of Technology, Wuhu 241003, China

## Abstract

E-commerce product recommendation system can help users to find their own products quickly from a large number of products. To address the shortcomings of the current e-commerce product recommendation system, such as low efficiency and large recommendation errors, we designed an intelligent recommendation system based on social awareness and mobile computing. The behavioral characteristics of the current e-commerce product recommendation system are analyzed; the e-commerce product recommendation system is built according to the data processing technology of mobile computing, and the key technologies of the e-commerce product recommendation system are designed. The test results show that the proposed system overcomes the shortcomings of the traditional e-commerce product recommendation system, speeds up the speed of users to find the products they really need from a large number of products, improves the accuracy of e-commerce product recommendations, and the error of e-commerce product recommendations is much lower than that of the traditional, which has higher practical application value.

## 1. Introduction

With the continuous development of information technology, logistics technology, network technology, and intelligent technology, the number and variety of goods on the Internet has increased dramatically. Goods have been stored in huge quantities, and at the same time, people are trading goods on the Internet more and more frequently, and many types of e-commerce management systems have emerged [1–3]. Among the e-commerce management systems, the e-commerce product recommendation system is one of the most important subsystems, directly affecting whether users can efficiently search for the e-commerce products they want. Therefore, the design and research of recommendation systems have been an important research direction in the field of e-commerce applications [4–6]. The traditional e-commerce product recommendation system uses a single computer to manage all user requests and product data, but with the increasing number of users and product data, the shortcomings of the single-computer model have become increasingly evident, mainly in the slow speed of the e-commerce product recommendation system, which makes it difficult to find the products that users really need within a short period of time [7–9].

The core task is to provide users with personalized product recommendation services by exploring the connection between users and products. Ultimately, achieving a win-win situation for both users and system owners [10, 11]. Large-scale e-commerce recommendation systems in the context of modern Internet applications are facing challenges in the following aspects: The data processing capacity of recommendation systems with a centralized architecture is limited. Stand-alone recommendation algorithms suffer from data processing scale limitations and processing efficiency problems [12]. In addition to the large number of users and products in large e-commerce systems, there are also many natural attributes of users and products, making it difficult to build accurate and effective models for high-dimensional users and products [13]. Business application requirements are often complex and variable, and user concerns vary for different application scenarios, so recommendation systems based on fixed models and parameters often lack flexibility [14]. Recommendation models are often strongly correlated with data characteristics and application scenarios, which dictates that recommendation systems must integrate a variety of complementary recommendation technologies. Algorithms and models of existing solutions are relatively homogeneous, making it difficult to meet the mainstream needs of mainstream users while taking into account their individual needs [15].

In order to overcome the shortcomings of the stand-alone e-commerce product recommendation system, some scholars have designed a distributed processing technology-based e-commerce product recommendation system. The distributed processing system relies on the Internet to unify the management of multiple stand-alone machines, which significantly improves the efficiency of the e-commerce product recommendation system compared to the stand-alone working mode, but there are some shortcomings in the distributed e-commerce product recommendation system, such as the recommendation efficiency is still difficult to meet the user's requirements for a large quantity, and the e-commerce product recommendation error rate is high [5]. Mobile computing is a fast processing system based on a distributed system, with the advantages of parallelism, distribution, and robustness, and has been successfully applied in many big data processing fields [16].

## 2. Related Technical Analysis

### 2.1. Comparison of the Main Recommended Technologies

The advantages and disadvantages of commonly used recommendation techniques, such as collaborative filtering, association rule mining, and knowledge-based empirical methods, are compared in Table 1.

### 2.2. Distributed Computing and Storage Technologies

Google's papers on distributed infrastructure have had a huge impact on the industry, with ideas such as MapReduce [5] and GFS [17] providing key references for distributed computing and storage, of which Hadoop is an open-source implementation [18]. Hadoop avoids time-consuming data transfer problems when dealing with large-scale data by using mechanisms for distributed data storage and migrating code rather than migrating data; it allows the system to recover from node failures by using mechanisms for moderate data redundancy.

## 3. Dynamic Community Segmentation Based on Mobile Behavioral Similarity

**Definition 1 .**

: Mobile behavioral characteristics. Mobile behavior characteristics reflect the spatial and temporal distribution of users' movements in different spatial locations within a given time interval [19]. In this paper, we choose the spatial frequency and length of stay of users as the portrayal of mobile behavior characteristics, which can be expressed as

(1) $$\begin{array}{c} o\left(w_{j},l_{i}\right)=\frac{f\left(w_{j},l_{i}\right)}{f\left(w_{j},l\right)}\times \frac{d\left(w_{j},l_{i}\right)}{d\left(w_{j},l\right)}, \end{array}$$

where *o*(*w*_*j*_, *l*_*i*_) represents the mobile behavioral characteristics of user *w*_*j*_ at a spatial location *l*_*i*_, and *f*(*w*_*j*_, *l*) represents the frequency of visits by user *w* at *f* and at all spatial locations *f*, respectively, and *d*(*w*_*j*_, *l*_*i*_) and *d*(*w*_*j*_, *l*) represent the length of stay of *W*, at *l*_*i*_ , and at all spatial locations *z*, respectively. The distribution of the characteristics of the movement behavior of user *W*, at all spatial locations, constitutes a *q*-dimensional vector (discrete spatial location-scale *q*) as

(2) $$\begin{array}{c} V\left(w_{j},l\right)=\left(o\left(w_{j},l_{1}\right),o\left(w_{j},l_{2}\right),\ldots ,o\left(w_{j},l_{q}\right)\right). \end{array}$$

The distribution of mobile behavioral features used in mobile user community segmentation is a relative value calculation. In other words, the characteristic distribution portrays the user's “preference” for different spatial locations. In practice, the absolute values of the spatio-temporal distribution of different users in different spatial locations are different, i.e. *f*(*w*_*j*_, *l*_*i*_) and *d*(*w*_*j*_, *l*_*i*_) are significantly different, which is the basis for the concept of mobile activity of users within a community.

**Definition 2 .**

: Mobile activity. Mobile activity is relative to the distribution of mobile behavioral characteristics, which are essentially relative values, while mobile activity is an absolute value [20]. Mobile activity is defined as the product of the cumulative frequency of visits and length of stay of a user *W*, at different spatial locations, expressed as

(3) $$\begin{array}{c} a\left(w_{j},l\right)=\overset{q}{\underset{i=1}{\sum }}f\left(w_{j},l_{i}\right)\times \overset{q}{\underset{i=1}{\sum }}d\left(w_{j},l_{i}\right). \end{array}$$

**Definition 3 .**

: Mobile spatio-temporal communities. Given a discrete time interval *c*_*i*_ and a dataset of historical movement trajectories of a set of users *w*, the set of users is divided into a finite number of communities based on the calculation of the characteristics of the movement behavior of different users at different time intervals *c*_*i*_ and different spatial locations is expressed as follows:

(4) $$\begin{array}{c} P=\left\{p_{1},p_{1},p_{2},\ldots ,p_{k}\right\}, \end{array}$$

where *p*_*i*_=(*w*_*i*1_, *w*_*i*2_,…, *w*_*ix*_), *w*_*ij*_ corresponds to the *i*th segmented community, and users within the same community have similar mobile behavioral profile distribution, while users within different communities have different mobile behavioral profile distribution [21]. The following section describes the process of dividing mobile communities in detail. Using the mobile behavioral profile formula, the preference profile of each participating user for different spatial locations can be derived *o*(*w*_*j*_, *l*_*i*_) , for each user *w*, the profile is calculated at different spatial locations, and the resulting preference profile is expressed in the form of a matrix as follows:

(5) $$\begin{array}{c} M=\left[\begin{array}{cccc} m_{11} & m_{12} & \ldots & m_{1q}\\ m_{21} & m_{22} & \ldots & m_{2q}\\ \vdots & \vdots & \; & \vdots \\ m_{n1} & m_{n2} & \ldots & m_{nq} \end{array}\right], \end{array}$$

where *m*_*j*,*i*_=*o*(*w*_*j*_, *l*_*i*_), the cosine similarity is calculated for any 2-row vector of matrix *M* by the following formula:

(6) $$\begin{array}{c} \cos\;\theta_{j1,j2}=\frac{\sum_{i=1}^{n}\left(o\left(w_{j1},l_{i}\right)\times o\left(w_{j2},l_{i}\right)\right)}{\sqrt{\sum_{i=1}^{n}\left(o{\left(w_{j1},l_{i}\right)}^{2}\right)}\times \sqrt{\sum_{i=1}^{n}\left(o{\left(w_{j2},l_{i}\right)}^{2}\right)}}, \end{array}$$

The similarity between users *w*_*j*1_ and *w*_*j*2_ in all spatial locations based on the distribution of their mobile behavioral characteristics is represented by cos  *θ*_*j*1,*j*2_. Based on this similarity, the *k*-means clustering algorithm is used to classify the *n* participating users into communities, resulting in seven different mobile communities. As mentioned above, the mobile activity calculation is used to identify a unique community organizer in each of the divided mobile communities *m* as the end-user super-user for task reception and data upload with the MCS platform, and as the task coordinator between different user subordinates within the community [22]. In order to indirectly group the spatial locations by communities, we use the average value of the spatial preference vector of all users in the community to represent the community's preference for spatial locations. If the community structure is *p*_*k*_={*w*_*i*1_, *w*_*i*2_,…, *w*_*ip*_}, then the community preference for spatial location *μ*(*p*_*k*_, *l*) is expressed as

(7) $$\begin{array}{c} \mu \left(p_{k},l\right)=\frac{1}{p}\overset{ip}{\underset{x=i1}{\sum }}V\left(w_{x},l\right)=\frac{1}{p}\overset{ip}{\underset{x=i1}{\sum }}\left[o\left(w_{x},l_{1}\right),\ldots ,o\left(w_{x},l_{n}\right)\right]. \end{array}$$

## 4. Merchandise Recommendations for Mobile Computing

The traditional e-commerce product recommendation system uses a single-computer model, where the user's e-commerce product tasks and related data are all stored on a single computer, and all work is completed on this computer, making the intelligent recommendation of e-commerce products quite time-consuming and unable to meet the current requirements of e-commerce product development [23]. Mobile computing introduces parallelism and task decomposition techniques on the basis of distributed processing systems, where a large-scale task is processed in pieces, resulting in many subtasks, each of which is carried out by one computer (node), so that the processing results of each subtask are obtained, and finally, the results of the subtasks are fused to obtain the final processing results, shown in Figure 1.

In an e-commerce product intelligent recommendation system, the recommendation algorithm is very critical, which directly affects the effect of e-commerce product intelligent recommendation. Therefore, this paper presents the specific design of the e-commerce product intelligent recommendation algorithm.

Let there be N users, which are denoted as User={*u*_1_, *u*_2_,…, *u*_*j*_,…, *u*_*N*_}, and all e-commerce products are denoted as  Item ={*i*_1_, *i*_2_,…, *i*_*j*_,…, *i*_*p*_}, and *p* denotes the total number of e-commerce products; there are *M* user tags, which can be denoted as Tag={*t*_1_, *t*_2_,…, *t*_*j*_,…, *t*_*M*_} so that the frequency of users clicking on e-commerce products and the corresponding tag values of e-commerce products describe the user characteristics, which are calculated as follows [24]:

(8) $$\begin{array}{c} V_{ut_{l}}={\text{tf}}_{\text{user rax}}\cdot {\text{idf}}_{{\text{user}}_{\text{tus}}}\cdot \left\{\frac{n_{ut_{l}}}{n_{ut}}\log\left(\frac{N}{N_{ul}}\right)\cdots \frac{n_{ut_{i}}}{n_{ut}}\log\left(\frac{N}{N_{n}}\right)\cdots \frac{n_{ul_{N}}}{n_{ut}}\log\left(\frac{N}{N_{ut_{N}}}\right)\right\}. \end{array}$$

Let *n*_*ut*_*i*__ and *n*_*ut*_ be the number of times a user uses *t*_*i*_ and the total number of tags used by a user respectively, then the frequency of tags and the popularity of tags to users are calculated as follows:

(9) $$\begin{array}{c} {\text{tf}}_{{\text{user}}_{l}ag}=\frac{n_{ut_{i}}}{n_{ut}},\\ {\text{idf}}_{{\text{user}}_{l}ag}=\log\left(\frac{n}{n_{ut_{N}}}\right). \end{array}$$

The feature vector describes the importance of e-commerce good and is calculated using the following metric:

(10) $$\begin{array}{c} V_{ut_{j}}={\text{tf}}_{{\text{item}}_{\text{ux}}}\cdot {\text{idf}}_{{\text{item}}_{\text{ta}}}\cdot \left\{\frac{n_{it_{l}}}{n_{it}}\log\left(\frac{P}{N_{it_{i}}}\right)\cdots \frac{n_{i_{i}}}{n_{it}}\log\left(\frac{P}{N_{i_{j}}}\right)\cdots \frac{n_{it_{H}}}{n_{it}}\log\left(\frac{P}{N_{it_{N}}}\right)\right\}. \end{array}$$

where tf_item_ux__ and idf_item_ta__ denote the frequency and importance of the use of the e-commerce good, respectively; *n*_*it*_*l*__ is the number of times e-commerce good *i* is used for the jth time; *n*_*it*_ denotes the total number of uses of e-commerce good *i*.

The user preference matrix for e-commerce goods is calculated as follows:

(11) $$\begin{array}{c} V_{uji_{k}}=\overset{M}{\underset{i=1}{\sum }}V_{uj}\times V_{i_{k}t} \end{array}$$

In which *u*_*j*_ ∈ *U*, *j*=1,2,…, *N*; *i*_*k*_ ∈ *I*, *k*=1,2,…, *P*.

The e-commerce product preference characteristics of users *u*_*j*_ are

(12) $$\begin{array}{c} V_{u_{j}}=\left(V_{uj,i},V_{uji},\ldots ,V_{uji_{k}},\ldots ,V_{u,i_{i}}\right), \end{array}$$

where *V*_*uji*_*k*__ is the preference level of *u*_*j*_ for e-commerce products. Based on the user's preference vector for e-commerce products, the user e-commerce product preference matrix is established as

(13) $$\begin{array}{c} V_{N\times P}=\left[\begin{array}{ccccc} V_{u_{1}i_{1}} & \cdots & V_{u_{1}i_{k}} & \cdots & V_{u_{1}i_{p}}\\ \vdots & \ddots & \vdots & \ddots & \vdots \\ V_{u_{j}i_{1}} & \cdots & V_{u_{j}i_{k}} & \cdots & V_{u_{j}i_{p}}\\ \vdots & \ddots & \vdots & \ddots & \vdots \\ V_{u_{N}i_{1}} & \cdots & V_{u_{N}i_{k}} & \cdots & V_{u_{N}i_{p}} \end{array}\right]. \end{array}$$

Similarity describes the degree of similarity between two e-commerce products, and intelligent recommendation algorithms obtain the similarity of e-commerce products based on cosine similarity [25]. The feature vector of an e-commerce product can be expressed as

(14) $$\begin{array}{c} I_{k}=\left(n_{k1},n_{k2},\ldots ,n_{ki},\ldots ,n_{kL}\right), \end{array}$$

where *n*_*ki*_ is the value of the *t*_*i*_-tagged e-commerce item *i*_*k*_ normalized. The full e-commerce product information can be described using the e-commerce product-specific vector matrix **I**_*k*×*k*_ as

(15) $$\begin{array}{c} I_{k\times k}=\left[\begin{array}{ccc} n_{11} & \cdots & n_{1k}\\ \vdots & \ddots & \vdots \\ n_{k1} & \cdots & n_{kk} \end{array}\right]. \end{array}$$

Cosine similarity between e-commerce products based on eigenvectors is expressed as follows:

(16) $$\begin{array}{c} \mathrm{sim}\left(i_{j},i_{k}\right)=\cos\left(I_{j},I_{k}\right)=\frac{I_{j}\cdot I_{k}}{\left|I_{j}\right|\times \left|I_{k}\right|}. \end{array}$$

(1) Let us divide an e-commerce product smart recommendation task and map each subtask to a corresponding mobile computation point via the map program [26]. (2) At each node, the user's preference matrix for the e-commerce product is calculated. (3) At each node, the similarity of e-commerce products is calculated and an e-commerce product similarity matrix is built. (4) Based on the user's historical search data for e-commerce products, each node searches the historical e-commerce products that user *u* has clicked on, and calculates the preference value between the user and the e-commerce product. (5) At each node, the preference values between users and e-commerce products are ranked, and the top N e-commerce products are selected as the intelligent recommendation results and the recommendation results of each node are obtained. (6) The recommendation results of each node are output to reduce, and the best *N* e-commerce products are finally recommended to the user through reduce fusion [27, 28].

The intelligent recommendation process of e-commerce products is shown in Figure 2.

## 5. Experimental Analysis and Testing

### 5.1. E-Commerce Product Datasets

To test the performance of the mobile computing-based e-commerce product recommendation system, an e-commerce management system with 50,000 e-commerce products and 2,000 users was selected as the test object. 80% of e-commerce product and user data were randomly selected as the training set, while the other data were used as the validation set. The performance of the e-commerce product intelligent recommendation system is evaluated by the accuracy and completeness rates, where the accuracy rate represents the accuracy of e-commerce product intelligent recommendation and the completeness rate represents the reliability of e-commerce product intelligent recommendation.

### 5.2. Comparison of Recommended Results

The accuracy and completeness rates of the e-commerce product intelligence recommendations are shown in Figures 3 and 4, respectively. It is clear from Figures 3 and 4 that the accuracy and completeness rates of the mobile computing-based e-commerce product intelligent recommendation are higher than those of the traditional e-commerce product intelligent recommendation. This is mainly because the e-commerce product intelligent recommendation algorithm in this paper takes into account users' preferences for e-commerce products, which improves the accuracy of the e-commerce product intelligent recommendation, and the reliability and stability of the e-commerce product recommendation are higher.

The recommendation time of the e-commerce product recommendation system is shown in Figure 5. As can be seen from Figure 5, the intelligent recommendation time for e-commerce products based on mobile computing has been significantly reduced, overcoming the shortcomings of the traditional e-commerce product intelligent recommendation system in terms of long recommendation times and low work efficiency, and helping users to find the e-commerce products they really need more quickly.

### 5.3. Social Perception Effect

This paper uses the WTD public dataset, which records approximately 11 weeks of communication data between 275 users with PDAs (personal digital assistants) and deployed APs on the UC San Diego campus, as experimental data. This dataset was used to validate the performance of the proposed group intelligence-aware social task distribution approach for mobile social networks. Due to the sparsity of different user data in the WTD dataset, 140 AP nodes are selected as spatial locations and 68 users are selected as participating users in this experiment. Distribution of mobile community behavioral features and the user connectivity network based on closeness is first tested.

The task execution effect, the number of task distributions, and the energy consumption of task recovery were tested by randomly generating 100–400 mobile group intelligence-aware tasks, with the spatial location of the tasks randomly selected from 140 AP points and the time interval randomly selected from 0 : 00 to 24 : 00. The relevant parameters are set as follows: the user fails to perform the task with a probability of 0.3, the community organizer respects a new performer with a probability of 0.5, and the task is passed through the social network with a probability of 0.5; in the case of passing the task, the person to whom the task is passed performs or refuses to perform the task with a probability value of their closeness. The energy consumption coefficient for data transfer via direct networks is set to 1, and the energy consumption for data transfer via opportunistic networks is set to 0.4. The specific distribution of the socially connected network in terms of closeness is shown in Figure 6.

Figure 7 shows a comparison experiment between the random distribution strategy and the traditional sequential distribution strategy, as well as an experiment with different intervention strategies after task execution failure, where vs is the number of group wisdom-aware tasks and *z* is the task completion rate. In the comparison between the random distribution strategy and the traditional sequential distribution strategy, there is no replacement of users for the failed task, and if the selected user does not appear in the specified spatial area on the second day at the corresponding time interval, the task fails. It can be seen from the figure that the proposed random distribution strategy significantly outperforms the traditional sequential distribution strategy.

Figure 8 shows the distribution statistics of the tasks under the task execution failure intervention experiment and the results of the perceptual data recovery energy simulation experiment, where B is the number of task distributions, *u* is the energy consumption statistics, and IV is the number of tasks. The statistics of the number of task distributions under the failed intervention experiment show that the number of distributions is lowest for the community-based distribution and the social intimacy-based user delivery, followed by the community-based distribution and the replacement within the failed user community, and the traditional “platform one user” full user reselection. The reason for this is that user delivery and distribution based on social intimacy has a high rate of task acceptance and execution. In addition to the above experiment, a questionnaire was conducted to simulate a real-life campus environment. This figure is generally consistent with the results of the WTD test. The reason for this is that the dynamic community segmentation based on spatio-temporal mobile behavior clusters users with similar mobile behavior so that suitable users can be searched for within a relatively small range of available users for replacement. The results of the perceived data recovery energy consumption simulation show that the optimal replacement strategy within the failed user community is, in order, social relationship-based intimate user delivery and distribution and the traditional “platform one user” full user reselection. The reason for this is that the optimal intracommunity replacement strategy maximizes the use of opportunistic mobile social networks for short-range communication and therefore consumes the least amount of energy, while the social relationship-based intimate user transfer and distribution comes second and the traditional “platform one user” full user reelection uses 3 G/4 G communication for data upload/download, which consumes the most energy. The energy consumption is the highest.

## 6. Conclusions

In order to overcome the shortcomings of the current e-commerce product recommendation system, this paper proposes a mobile computing-based e-commerce product recommendation system. Firstly, to address the shortcomings of the current e-commerce product recommendation system based on the stand-alone working mode, such as low efficiency and slow speed, the mobile computing working mode was introduced to decompose the e-commerce product recommendation task and carry out distributed and parallel processing; secondly, to address the problem of large recommendation errors in the e-commerce product recommendation system, the e-commerce product intelligent recommendation system integrates the user's preference for products. The results show that this paper's e-commerce product intelligent recommendation system works efficiently and has high accuracy in recommending e-commerce products, which can provide valuable reference advice for users when conducting e-commerce product transactions.

## Figures and Tables

**Figure 1:** Working principle of e-commerce product recommendation system for mobile computing.

**Figure 2:** Intelligent recommendation process for e-commerce products.

**Figure 3:** Recall of e-commerce product intelligence recommendation system.

**Figure 4:** Completeness rate of intelligent recommendation systems for e-commerce products.

**Figure 5:** Recommendation time of an intelligent recommendation system for e-commerce products.

**Figure 6:** Social connection network based on intimacy.

**Figure 7:** MCS task distribution experiment I.

**Figure 8:** MCS task distribution experiment II.

**Table 1:** Comparison of the main recommended technologies.

	Advantage	Shortcoming
Collaborative filtering technology	Discover new and different interests and do not depend on domain knowledge. With the passage of time and the accumulation of data, the effect is getting better and better. The recommendation process has a high degree of personalization and automation and can deal with complex unstructured objects	There are typical problems such as scalability, sparsity and cold start, and the recommendation quality depends on the historical data set
Association rule mining	Can discover new and different points of interest, independent of domain knowledge	Rule extraction is difficult and time-consuming, and the degree of personalization is low
Knowledge experience-based approach	It can consider nonproduct attributes, reflect user needs, and make up for the lack of user knowledge and experience	Knowledge and experience are difficult to obtain, and recommendation is static

## Data Availability

The datasets used during the current study are available from the corresponding author on reasonable request.
